# Visual Object Tracking Algorithm Based on Biological Visual Information Features and Few-Shot Learning

**DOI:** 10.1155/2022/3422859

**Published:** 2022-03-03

**Authors:** Dawei Zhang, Tingting Yang

**Affiliations:** School of Computer and Artificial Intelligence, Zhengzhou University, Zhengzhou, Henan 450001, China

## Abstract

Eye tracking is currently a research hotspot in the territory of service robotics. There is an urgent need for machine vision technique in the territory of video surveillance, and biological visual object following is one of the important basic research problems. By tracking the object of interest and recording the tracking trajectory, we can extract a structure from a video. It can also analyze the abnormal behavior of groups or individuals in the video or assist the public security organs in inquiring and searching for evidence of criminal suspects, etc. Moving object following has always been one of the frontier topics in the territory of machine vision, and it has very important appliances in mobile robot positioning and navigation, multirobot formation, lunar exploration, and intelligent monitoring. Moving object following has always been one of the frontier topics in the territory of machine vision, and it has very important appliances in mobile robot positioning and navigation, multirobot formation, lunar exploration, and intelligent monitoring. Moving object following in visual surveillance is easily affected by factors such as occlusion, rapid object movement, and appearance changes, and it is difficult to solve these problems effectively with single-layer features. This paper adopts a visual object following algorithm based on visual information features and few-shot learning, which effectively improves the accuracy and robustness of tracking.

## 1. Introduction

With the rapid expand of computer picture capabilities and technologies, and the improvement of the cost-effectiveness of a large number of digital picture equipment, vision systems have been widely adopted by mobile robots [1]. Computer vision is the most common method for humans to obtain environmental data via computers. Understanding the visual attention mechanism allows humans to process salient information in complex scenes quickly and efficiently, while masking and ignoring nonsalient regions autonomously. Machine learning is a century-old technology that is destined to thrive in the age of data. Machine learning's [2] advantage is that it can automatically analyze and process unknown data by mining and learning from existing data, reducing the need for human resources to the greatest extent possible. Scholars in the United States and abroad have conducted extensive and in-depth research on object recognition, object following, navigation, monitoring, and other technologies based on robot vision [3]. Machine vision's primary goal is to enable computers to mimic human thinking activities, obtain information from visual sensors to gain an understanding of the environment, and finally realize the computer's autonomous adaptation to the environment [4]. Researchers in the United States and abroad are using computers to create a visual attention model that simulates the human attention mechanism and incorporates it into the processes of object detection [5], object recognition, and moving object following, in order to bring the object processing process closer to the human cognitive mechanism and improve the algorithm's performance. This area of research has become one of the most active in the field of pattern recognition. Video image data contains the most information of all the data circulated or saved on the Internet, but extracting it is extremely difficult. According to the number of cameras mounted on the robot, monocular vision and stereo vision can be distinguished. Computer vision is a multidisciplinary field that includes computer science, physics, physiology, psychology, artificial intelligence [6, 7], semaphore processing, and applied mathematics.

The traditional mean-shift algorithm is based on the matching search process of the object color feature histogram, but the color features are not sensitive to noise and occlusion. So many surveillance cameras will generate massive amounts of surveillance video data every day, and these surveillance videos contain useful information that can be used to cardinaltain social stability, travel safety, and traffic guidance. Although the traffic police department has the right to use these surveillance cameras, there are many problems in analyzing these surveillance videos solely by the human eye. The cardinal difficulty in the research of moving object following algorithm in complex scene is the robustness and accuracy of the tracking algorithm. Monocular vision is inferior to stereo vision in terms of depth extraction, but it is comparable to stereo vision in terms of feature extraction and matching, and it avoids the problem of stereo vision binocular objecting, improves real-time performance, and has a simple structure. Machine vision technology has now penetrated many areas of the national economy, including aerospace, remote sensing and telemetry, medical aided diagnosis, map drawing, industrial security, multimedia communications, intelligent robots, and other areas. Simply relying on the human eye to analyze surveillance video will consume a significant amount of human resources, and the human eye has a blind spot and causes visual fatigue, making it impossible to maintain a long-term focus on the surveillance video [8]. This shows that there is an urgent need for machine vision technique in the territory of video surveillance [9]. With the expansion of machine vision, vision-based object following technique has become a hot spot in engineering and academia. Moving object tracking refers to the detection, identification and sports tracker objects in the video, and obtaining some motion parameters of the moving objects, such as speed, position, acceleration, and motion trajectory, so as to achieve higher-level processing and analysis [10]. The behavior of the object is understood and prepared to complete a specific task.

Object recognition is the foundation of tracking in an eye tracking system, and accurate object recognition is required for effective tracking [11]. This paper uses a visual object following algorithm based on visual information features to achieve accurate object following in complex backgrounds while overcoming partial occlusion and background fusion interference.

## 2. Related Work

The Harris affine detector was proposed in [12], which combines the Harris corner detector and the Laplace equation to ensure that the detected features are scale-invariant. Reference [13] proposes an edge-based area detector that constructs parallelograms around Harris corners using curved and straight edges. The most stable extremum region detector, which is a watershed-like approach, is proposed in [14]. To achieve effective multiview matching, [15] proposed using complex filters to generate kernel functions. Reference [16] proposes phase-based local features to improve lighting change robustness. Literature [17] proposed PCA-SIFT, which uses principal component analysis to simplify the SIFT descriptor, standardize the gradient region, and achieve fast matching and invariance under image distortion. Reference [18] proposes a rotation-invariant feature transformation, which divides each standard circle into a series of concentric circles, and each concentric circle is associated with a gradient orientation histogram. Reference [19] proposed that the gradient position and orientation histogram is an extension of the SIFT descriptor. Similar to PCA-SIFT, GLOH also reduces the dimensionality of descriptors through principal component analysis. Literature [20] proposed four color descriptors, namely, RGB histogram, hue histogram, vertex angle histogram, and spherical angle histogram. Reference [21] proposed a global positioning way for mobile robots based on monocular vision. Reference [22] proposes a hierarchical real-time localization and map creation way for mobile robots based on an active closed-loop strategy.

In this paper, a visual object following algorithm based on visual information features is adopted, which has good real-time performance, accuracy, and practicability. It combines sequential detection mechanism, binocular disparity information, and binocular vision calibration model to complete object recognition and localization and can achieve good tracking accuracy.

## 3. Research on Visual Object Tracking

### 3.1. Robot Vision

The identification and tracking module, the robot control module, and the robot platform make up the vision system [23]. Since their first appearance in the 1960s, robots have gone through three historical stages around the world. With the rapid growth of the robot industry at home and abroad, as well as significant progress in the field of artificial intelligence, the role of robots in human life has become increasingly important in recent years. Eye tracking is a hot topic in the field of machine vision as well as an important research direction in the field of intelligent mobile robots. With the advancement of science and technology in recent years, an increasing number of products have begun to use machine vision-related technologies, and an increasing number of scholars have devoted themselves to picture-related territories for research and expansion [24]. Algorithms started to evolve into useful devices. The advantages of visual semaphores include a wide range of semaphore detection and a large amount of data acquisition. Eye tracking has become one of the cardinal expansion orientations in the field of robotics, thanks to the rapid expansion of picture technique and computer processing capability in recent years. Robots currently perform the majority of their work by following preprogrammed instructions to perform repetitive and specific tasks [25]. The robot must be reprogrammed to adapt to the new operating environment if the operating environment changes. Machine vision is booming, and it is providing a lot of technical support for robot technique improvement. Visual servosystems have recently emerged as a key research topic in the field of robot control. One of the key technologies of mobile robot vision is real-time sports tracker objects [26]. The basic principle block diagram of maneuvering object following is shown in Figure 1.

In order to achieve fast and effective tracking of the object, this paper proposes an improved eye tracking algorithm for mobile robots, which is based on the mean-shift algorithm, uses color features as the basis for eye tracking, and introduces Kalman filtering to predict the iterative window. The identification and tracking module adopts the improved Camshift algorithm and the way of Kalman filter [1] to identify and track the selected tracking object; the robot control module cardinally completes functions such as sending robot control instructions. With the continuous expansion of domestic and foreign scientific and technological level, computer technique, sensor technique, artificial intelligence, and robotics have developed rapidly, so that the application of robots is no longer limited to the industrial territory. Military territories such as territory, underwater, and space, as well as indoor environments such as hospitals and exhibition halls, have also been included in the application within the range [27]. At the same time, in recent years, the state has proposed the establishment of a smart city and a safe city where all things are perceived, connected, and intelligent, so that the domestic security industry can gain opportunities for rapid expansion, so that machine vision research continues to be hot, and robots can be obtained through the vision system and a large amount of information and then through the information processing and finally making a decision.

Eye tracking technique is an important research orientation in the territory of intelligent mobile robots, and it is also a hot issue in the territory of machine vision. Vision-based mobile robot tracking techniques have advanced rapidly in the last two decades. The robot's recognition and sports tracker objects require segmenting the image sequence obtained by the vision sensor into moving objects in the time do cardinal, as well as modeling, recognizing, and tracking these objects in the time do cardinal. The research on the robot with the object detection function can give the robot the ability to perceive the environment and perform servocontrol in response to changes in the environment. The visual servosystem completes the acquisition of visual image information through the camera during the robot control process, and the robot's function to obtain information from the outside world is realized. A mobile robot's intelligence is based on its ability to coordinate with external objects such as the environment and people. The vision system is crucial in this regard. A laptop and a control board comprise the robot platform. The eye tracking software is run on the laptop. The control board is in charge of driving the motor and gathering sensor data. The vision system can provide a wealth of information to the intelligent mobile robot, such as position and motion parameters, so that it can correctly perceive itself. Make the best decisions about your own behavior and the work environment in which you live.

### 3.2. Vision Based Object Tracking

#### 3.2.1. Object Recognition Based on Local Features

Object recognition has been widely used in medical diagnosis, military technique, security detection, and other domains as an important research orientation in the field of picture and pattern recognition. Image understanding, automatic image segmentation, moving object following, and scene understanding are all built on this foundation. Traditional object detection and tracking algorithms typically only use the image's underlying visual features to construct object descriptors in order to obtain a description of the object's appearance for object detection and tracking and obtain the object's location information in order to realize the object's detection and tracking. Machine vision research's main goal is to use computers to simulate and realize visual functions similar to those performed by the human eye, such as object, scene, and motion detection, as well as three-dimensional reconstruction. The most important way for humans to obtain external information is through their vision system, and object recognition is a key topic in the field of machine vision and pattern recognition, which has a wide range of potential applications. Long-distance object recognition is difficult due to the image's complex background and the object's small number of pixels. Object detection is a hotspot of machine vision research, with applications in image retrieval, intelligent transportation, intelligent video surveillance, advanced human-computer interaction, and other areas. However, existing object detection methods have significant drawbacks, and a high-precision, high-efficiency, and high-robustness object detection algorithm in the field of machine vision is still urgently needed.

Common moving object detection ways can be divided into three categories: interframe difference way, optical flow way, and background subtraction way. Feature extraction is a key technique in object recognition, which plays a decisive role in the final result of recognition. Aiming at the problem of viewing angle, scale, and brightness condition changes in automatic object recognition, and the disadvantage of low recognition rate of local features is when the viewing angle and brightness change are large. The images generated in real scenes often have many complex situations such as changes in illumination intensity, object scale scaling, different imaging perspectives, object occlusion, and redundant background interference [28]. A problem in the actual process, in addition to the pose, scale, rotation, and translation changes of the object itself, is that there are also challenges such as illumination changes, complex backgrounds, and object occlusion. Recognition of objects/objects is one of the important orientations and can be divided into 3 categories according to the generality of the recognition objects: recognition of specific objects (the same thing), recognition of a series of objects (such as aircraft, ships, people, and face), and object recognition in general (and the ability to spot any object). In national defense construction, object recognition is a key technique in training, reconnaissance, and defense systems. For example, defense systems mostly use object recognition technique to track, identify, and guide missiles on mobile military objects. Robot is a multidisciplinary application technique that integrates machinery, computer, automatic control, etc.

At present, the research in this territory is active and the application is increasingly widespread. Object detection has become a challenging problem due to the uncertainty of the appearance shape of different objects, the complexity of the application scene, the mutual occlusion between objects and between objects and the background, etc. Neurophysiological studies have revealed in recent years that, in the primitive visual cortex of mammals, a sparse coding strategy is used. The human visual system can break down objects into a variety of small, meaningful pieces and use this information to identify the object robust to occlusion and pose changes, in addition other excellent properties. The object detection method based on local features has quickly become a research hotspot at home and abroad. The purpose of the local feature synthesis link is to combine a large number of local features into a single feature, resulting in more reliable features for the classifier design. The detection algorithm based on joint features is a new trend in current expansion because a single feature mode cannot accurately detect the object.

#### 3.2.2. Object Description and Data Fusion in Visual Tracking

In recent years, with the rapid expansion of computer technique, computers no longer have simple data processing functions, but have become more and more intelligent. Target tracking is a research topic with extensive practical application significance in military and civilian territories. To realize the effective and accurate identification and tracking of the object under the difficult problem of tracking, the key is how to describe the tracking object adaptively and accurately model the tracking object. Since the expansion of object following technique in the middle of the last century, it has been widely used in various territories such as industrial robots, video surveillance, and missile interception. Intelligent video surveillance is a new type of video surveillance technique gradually developed by introducing relevant research results in machine vision into traditional video surveillance. Since the birth of the first robot in 1959, robot technique has made great progress and expansion and has become a comprehensive cutting-edge science that integrates machinery, electronics, computers, control, sensors, semaphore processing, and other disciplines. The role of robot object tracking in indoor environment is becoming more and more important.

Artificial intelligence technique subverts the traditional way of thinking of human beings, so that human beings have a new understanding of artificial intelligence. The key to effectively complete the corresponding tasks of the UAV lies in the various information provided by the external sensors mounted on it. The sensors usually used are mostly sonar, inertial navigation systems, barometers, magnetometers, etc., relying on Global Positioning System. The so-called machine vision is a simulation of biological vision using computers and related equipment. The origin of object following can be traced back to 1937, that is, on the eve of World War II, when a tracking radar named SCR-28 appeared for the first time, and its appearance marked that object following officially entered people's territory of vision. Intelligent video surveillance automatically comprehends image content without human intervention. When the individual or group behavior is abnormal, the alarm can be timely, so that the video surveillance can get rid of the dependence on the all-weather manual supervision. Intelligent robots can acquire, process, and recognize a variety of information and autonomously complete more complex tasks.

Continuous and stable sports tracker objects can not only obtain the position information of the current moving object, but also help to conduct a more in-depth analysis of the moving state of the object, so as to achieve precise positioning and intelligent control of moving objects. Guidance, vehicle navigation, human-computer interaction, and other territories have broad application prospects and great economic value. Detecting objects in videos solely using still image object detection methods is insufficient because they cannot handle useful information such as temporal and contextual information. Sensors commonly used are slightly insufficient for obtaining more accurate information about the surrounding environment or objects. When faced with this problem, applying machine vision techniques and visual sensors to UAVs, which have developed rapidly in recent decades, is an effective way to compensate for the shortcomings of traditional common sensors. Computer vision is the use of cameras or computers to simulate the capture of external objects instead of human eyes, and machine vision can process visual information according to the characteristics of computer systems through processing to enable people to understand intuitively. The technique of target tracking has grown in importance as a field of study. It has been widely concerned and applied, and it plays a pivotal and important role in industry, military affairs, and everyday life.

## 4. Visual Object Tracking Algorithm Based on Visual Information Features

### 4.1. Object Recognition Based on SIFT Features

Images have become a necessary means for humans to obtain information from the outside world as society has progressed and information technology has rapidly expanded, and the use of computers to process images to obtain information of interest to humans has become a hot research topic. Many vision appliances use image matching as a key technique. In this paper, the video stream monitored by the camera is used to control the specific object. Finally, key frame image matching is required, and the effect of matching has a direct impact on the effect of subsequent analysis and processing. Detecting and tracking moving objects has always been a challenge in video surveillance systems. Many scholars have conducted extensive research on this issue in recent years, but it remains a difficult subject. At the moment, the most common method of background modeling is to update the background statistics, with single Gaussian models, mixed Gaussian models, and their improved algorithms being the most commonly used methods. By modeling the surveillance area scene's mixed Gaussian background in the video stream, each pixel of the background image is modeled by a mixed Gaussian model made up of K Gaussian distributions:

(1) PXi=∑i=1Kωi,t•μXt,ηi,t,Σi,t,Xt=xtr,xtg,xtb,ηi,t=μi,tr,μi,tg,μi,tb.

Before extreme point detection, the original image is preprocessed to remove noise. Then, an upscaled linear interpolation is performed on the image. Next, construct Gaussian pyramid and DOG pyramid to filter the image.

The scale space *L*(*x*, *y*, *σ*) is established as follows:

(2) $$\begin{array}{c} L\left(x,y,\sigma \right)=\left(G\left(x,y,\sigma \right)\right)*I\left(x,y\right). \end{array}$$

Here *I*(*x*, *y*) is the original image, *σ* is the standard mean square error, ^*∗*^ is the convolution operation, and *G*(*x*, *y*, *σ*) is the scale-variable Gaussian.

(3) $$\begin{array}{c} G\left(x,y,\sigma \right)=\frac{1}{2\pi \sigma^{2}}e^{-\left(x^{2}+y^{2}\right)/\left(2\sigma^{2}\right)}. \end{array}$$

The DOG filter is defined as follows:

(4) $$\begin{array}{c} D\left(x,y,\sigma \right)=L\left(x,y,k\sigma \right)-L\left(x,y,\sigma \right). \end{array}$$

Here *k* is a constant.

At the moment, most commercial object recognition systems use a template-matching approach. This method, however, places strict limitations on the object's position and brightness, and the matching effect is not ideal when the object's rotation, scaling, brightness, or 3D pose change. Many feature points are extracted by the traditional SIFT algorithm during the feature extraction stage, lengthening the recognition process and increasing the false matching rate. The camera is mostly stationary in most practical scenes, creating a “static background.” However, as technology advances and the need to cut costs grows, the camera must move more and more to achieve continuous sports tracker objects and thus expand the monitoring range. The work-based object recognition technique is a type of pattern recognition that has both theoretical and practical applications. Despite the fact that significant progress has been made in this research, there are still numerous obstacles to overcome. Moving object detection and tracking has become commonplace in areas such as traffic management, image analysis and processing, video conferencing, and bank surveillance. The object position, including the object's pose change, can be accurately identified using the method described in this paper, and the recognition effect is good as shown in Figures 2, 3, and 4.

Because of its excellent matching performance, the matching algorithm based on multiscale space has attracted the attention of many researchers in recent years, and it has achieved great results by applying it to various appliances. A SIFT extreme value detection algorithm based on significant edge constraints is used to detect the bottom of the pyramid in the research on the identification of specific building areas in remote sense images, based on the characteristics of large territory of view remote sense images with large imaging range and complex scenes, combined with the geometric characteristics of the building area to be identified. To obtain binary images, adaptive threshold segmentation of images is used. To meet the requirements of object recognition, the SIFT feature matching algorithm needs to be improved according to the specific scene. Because image feature matching and object recognition have a lot in common, it is a good idea to use feature matching to achieve object recognition. The entire background changes as the camera moves, making it more difficult to detect moving objects against a static background. The flowchart of the background subtraction way is shown in Figure 5.

The identification of a specific object belongs to static image matching. The feature point extraction of the image and the calculation of the minimum distance are used as the cardinal ways to find the difference between the pixels of the same scene projected to the specific object image in the two images of the specific object and the given scene. Correspondence: in the past, object recognition technique based on image features has achieved good results in specific territories, and the emergence of feature extraction algorithms has brought a new idea and way to object recognition research. The detection of moving objects can obtain the relevant information of the object objects in the sequence images. By extracting the moving objects and their related information in the sequence images and segmenting and analyzing the objects, it lays the groundwork for the later part of the object following. In video surveillance system, moving object detection is the basis and premise of moving object tracking, which plays a very important role in many territories and is of great significance to video surveillance and so on.

### 4.2. Tracking Algorithm Analysis

After decades of unremitting efforts of scholars, moving object detection and tracking technique has made great progress. However, due to the complexity of the application environment of the eye tracking system, such as illumination, occlusion, and other factors and the diversity of the object itself, it brings great difficulties to the object detection and tracking technique. In terms of accuracy, the appearance of the background and the object in the video image may change at any time, and it is difficult for the existing picture algorithms to accurately identify the object in the image sequence. Computer vision is a highly comprehensive subject with many interlaced disciplines. Its content involves many disciplines such as picture, artificial intelligence, pattern recognition, and neural network. The image is sent to the computer for related processing. Among the many research orientations of machine vision, eye tracking has always been one of the most important research hotspots at home and abroad and belongs to the middle-level processing part of machine vision. Its purpose is to process, detect, locate, and track objects of interest in the video sequence captured by the camera. Robotics is a combination of theoretical and scientific research achievements in various territories such as computer technique, automatic control, communication, machinery, and artificial intelligence. As robots play an increasingly important role in the current human economic expansion and technological progress, the application territories of robots continue to expand, the tasks faced by robots are becoming more and more complex, and the working environment is becoming more and more complex.

The research of machine vision has two meanings. One is to meet the requirements of artificial intelligence appliances, i.e., to use computers to realize the requirements of artificial vision systems. These findings can be installed on a variety of robots, giving them the ability to “see.” Second, the machine vision model's research findings can help us better understand and study the human visual system's mechanism, as well as the human brain's mechanism, which is also important to know about. Picture algorithms generally model the appearance and background of the object in the image based on pixel points, which has the characteristics of a large amount of calculation, especially when faced with a large number of images to be processed, and the real-time performance of the object following algorithm can be solved significantly. Due to some flaws in human beings, they are unable to meet the current needs in terms of time and work intensity in such a big data era that today's society is experiencing. As the times demand, the intelligent video surveillance system emerges, successfully defeating traditional surveillance systems as well as human beings. The intelligent video surveillance system converts the traditional passive monitoring strategy of “forensics after the event” into an intelligent and active monitoring mode that incorporates “real-time monitoring and prior prevention.” For incremental subspace learning in this paper, two eigenvectors are used. Figures 6 and 7 show how this works.

The trend of each monitored object and the interaction between the monitored objects can be obtained by tracking in the intelligent monitoring system, allowing for more in-depth analysis of the monitored object's behavior and the detection of specific events. In the realm of intelligent transportation, vehicle and pedestrian tracking can improve the degree of automation in traffic accident detection, as well as enabling judgment of vehicle driving states, which can then be used to understand road traffic conditions and provide intelligent traffic guidance. It is becoming increasingly difficult to meet the task requirements due to the limitations of a single robot's movement and perception abilities. The collaborative theory of heterogeneous robots was born out of this situation. People give multiple heterogeneous robots the ability to collaborate with one another, expand the robot's scope of action, and improve the robot's ability to complete complex tasks. Many researchers have conducted fruitful research on the eye tracking problem and proposed many tracking algorithms in order to achieve the goal of intelligent motion perception. They have proposed a number of solutions to the eye tracking issues. Through the collaboration and cooperation of multiple heterogeneous robots, the system can integrate all individual resources, and the entire system has parallelism in terms of space, time, information, and task execution. Improve the efficiency of processing tasks, thereby improving the completion rate of tasks and enhancing the robustness of the system.

## 5. Conclusions

Computer science, machine vision, picture, pattern recognition, artificial intelligence, automatic control, and other theories have come together to form mobile robot navigation and positioning. Through correlation filtering operations, the affine transformation information experienced by the object during motion can be extracted. A visual object following algorithm based on visual information features is proposed in this paper. The algorithm uses pixel-level object background segmentation to obtain a rough object distribution template and then uses that information to perform threshold-adaptive voting decision classification in the superpixel area to eliminate noise interference and obtain a more accurate object distribution. Video object tracking combines machine vision, image processing, pattern recognition, and artificial intelligence. It is a relatively new research approach. In recent years, it has attracted more and more researchers' interest. However, despite the extensive use of video tracking, there are still a number of issues that need to be investigated further.

## Figures and Tables

**Figure 1:** Basic principle block diagram of maneuvering object following.

**Figure 2:** The relationship between the number of intermediate layers and the number of extreme points.

**Figure 3:** Relationship between the number of feature points and object parameters.

**Figure 4:** The relationship between the number of feature points and the changing parameters.

**Figure 5:** Flowchart of background subtraction way.

**Figure 6:** Center distance error 01.

**Figure 7:** Center distance error 02.

## Data Availability

The data used to support the findings of this study are included within the article.
